# Downregulation of LHPP Expression Associated with AFP Acts as a Good Prognostic Factor in Human Hepatocellular Carcinoma

**DOI:** 10.1155/2021/1971048

**Published:** 2021-08-25

**Authors:** Xu Chao, Wei Zhang, Jieqiong Wu, Xuesong Feng, Hailong Shi, Luyan Zhao, Haiyu Shen, Chao Jiang

**Affiliations:** ^1^The Second Affiliated Hospital of Shaanxi University of Chinese Medicine, Xianyang 712000, China; ^2^The College of Basic Medicine Sciences, Shaanxi University of Chinese Medicine, Xianyang 712046, China; ^3^The Second Affiliated Hospital of Xi'an Medical University, Xi'an, Shaanxi 710038, China

## Abstract

**Background:**

Phospholysine phosphohistidine inorganic pyrophosphate phosphatase (LHPP) serves as a tumor suppressor in hepatocellular carcinoma (HCC), but the correlation between the expression of LHPP and the clinical parameters of oncogenic progression is still not well defined. This study is to reveal the correlation between the expression of LHPP in HCC and their clinical parameters.

**Methods:**

Immunohistochemical analysis was used to assess the correlation between the expression of LHPP and the clinical parameters of HCC. Expressions of LHPP in HCC tissues and cultured HCC cells were detected by Western blot and quantitative real-time polymerase chain reaction (qRT-PCR). LHPP, gamma-glutamyl transferase (GGT), and *α*-fetoprotein (AFP) expression levels in blood or HCC tissues were detected by enzyme-linked immunosorbent assay (ELISA). The Spearman rank correlation coefficient was used to evaluate the correlation of the expression of LHPP and the clinical index of HCC. Correlation of survival and expression of LHPP were analyzed using the Kaplan-Meier method and the log-rank test.

**Results:**

Expressions of LHPP in HCC tissues were significantly downregulated than their paired adjacent normal tissues. A significant positive correlation was found between the cytoplasm and nuclear expression of LHPP in both HCC and their paired adjacent normal tissues. The expression of LHPP negatively correlated with the levels of GGT in the cytoplasm of adjacent tissues and with the AFP level in the nucleus of HCC cells. Relative levels of LHPP in HCC tissues were markedly lower than those of the paired adjacent normal tissues. Relative levels of LHPP in LO-2 cells were higher than those of HepG2, BEL-7404, and SMMC-7721 cell lines. The overall survival and DSF survival of patients with the high expression of LHPP were much higher than those with the low expression of LHPP in paired adjacent normal tissue.

**Conclusions:**

LHPP is associated with the AFP level and acts as a good prognostic factor in HCC.

## 1. Background

Liver cancer was predicted to be the sixth most commonly diagnosed cancer and the fourth leading cause of cancer death worldwide in 2018, with about 841,000 new cases and 782,000 deaths annually [1]. In China, liver cancer is a common primary cancer in adults and a malignant tumor due to its high morbidity. It is also the second leading cause of cancer mortality [2, 3]. Invasion and intrahepatic metastasis are the main factors leading to poor prognosis of patients with hepatocellular carcinoma (HCC) [4]. Detecting the molecular mechanism of hepatocellular carcinoma might have a significant value in diagnosing and treating HCC [5].

LHPP encodes an enzyme known as phospholysine phosphohistidine inorganic pyrophosphate phosphatase (LHPP), which was originally purified from swine brain tissue [6]. Deregulated histidine phosphorylation has been found in various diseases [7]. LHPP gene variation is associated with the oral cavity and pharyngeal cancer [8]. LHPP may interact with serotonin receptor 1A (Htr1a) in the pathogenesis of major depression [9]. Patients with major depressive disorder having LHPP rs35936514 CT/TT genotype have increased activity in certain brain regions [6]. Recently, it has been reported that LHPP plays an essential role in inhibiting human HCC progression by regulating the phosphatidylinositol-3-kinase/protein kinase B (PI3K/Akt) signaling pathway [10]. LHPP serves as a tumor suppressor in liver cancer, and the loss of the expression of LHPP is associated with reduced survival in HCC [11, 12]. However, the correlation between the expression of LHPP and the clinical parameters of HCC in oncogenic progression is still not well defined.

This study is aimed at exploring the expression of LHPP in HCC and evaluating the correlation between the expression of LHPP and the clinical parameters of HCC. The findings might provide a new insight to improve the prognosis of patients and the survival rate of patients with HCC.

## 2. Methods

### 2.1. Materials

HepG2, BEL-7404, SMMC-7721, and LO-2 cells were purchased from the National Collection of Authenticated Cell Culture (Shanghai, China). RPMI-1640 media and fetal bovine serum were purchased from Gibco Co., Ltd. (NY, USA). Mouse anti-human *β*-actin and LHPP were purchased from Santa Cruz Biotechnology, Inc. (CA, USA). Human alpha-fetoprotein (AFP) and ELISA Kit were purchased from Abcam Biotechnology, Inc. (Shanghai, China). A GGT Activity Assay Kit was purchased from Amy Jet Scientific, Inc. (Wuhan, China).

### 2.2. Patients and Specimens

Two tissue microarrays (TMAs) of HCC samples were used to assess the correlation between the expression of LHPP and the clinical parameters of HCC. One was a survival liver cancer tissue chip (HLivH180Su14, Shanghai Outdo Biotech, Shanghai, China), which included 90 liver cancer and paired paracancerous samples with death and recurrence information and followed up for 3.8-4.6 years. The other was the HCC tissue microarray (HLivH060CD03, Shanghai Outdo Biotech), which included 2 normal liver specimens, liver samples of 6 patients with cirrhosis, 17 primary tumors and paired adjacent cancer samples (3 cases with distal normal liver tissue), and 15 liver cancer metastases cases. Conventional clinicopathological variables, including gender, age, hepatitis history, liver cirrhosis, AFP, GGT, tumor number, size, encapsulation, differentiation, vascular invasion, stage, therapy, and status, were recorded and are displayed in Table 1.

Five liver cancer and paired paracancerous samples used for WB and qRT-PCR experiments and the blood used for enzyme-linked immunosorbent assay (ELISA) come from the pathology department of Xijing Hospital of Air Force Military Medical University.

### 2.3. Cell Culture

HepG2, BEL-7404, SMMC-7721, and LO-2 cells were obtained from the National Collection of Authenticated Cell Culture (Shanghai, China). All cells were cultured in RPMI-1640 medium supplemented with 10% (*v*/*v*) heat-inactivated fetal bovine serum, 100 *μ*g/mL streptomycin, and 100 U/mL penicillin. The cultures were maintained at 37°C in a humidified atmosphere of 5% CO_2_. Cells in the exponential growth phase were used for all experiments.

### 2.4. Immunohistochemical Analysis

Immunohistochemical analysis was employed to detect the differential expression of LHPP in HCC tissues and paired adjacent normal tissue. Briefly, the sections were dewaxed, hydrated, and washed. After the neutralization of endogenous peroxidase and the microwave antigen retrieval, the slides were preincubated with blocking serum and then incubated overnight with the mouse anti-human LHPP monoclonal antibody (1 : 500) at 4°C. Subsequently, the sections were serially rinsed, incubated with second horseradish peroxidase- (HRP-) labeled anti-mouse antibody, and treated with horseradish peroxidase-conjugated streptavidin. The reaction products were visualized with 3,3-diaminobenzidine tetrahydrochloride and counterstained with hematoxylin after washing with phosphate-buffered saline.

The staining intensity was observed by two pathologists for immunohistochemical analysis. The scoring in detail was as follows: negative for 0, “+” for 1, “++” for 2, and “+++” for 3. The positive staining rate according to the proportion of positively stained cancer cells was defined as follows: “negative” for 0, “1%-20%” for 1, “21%-40%” for 2, “41%-60%” for 3, “61%-80%” for 4, and “81%-100%” for 5. The total score was the product of “dying intensity” score and “dying positive rate” score.

The HCC tissues and their paired adjacent normal tissues were grouped separately because the expression of LHPP in cancer tissues was significantly lower than that in adjacent tissues. In HCC tissues, the total LHPP expression score ≤ 1.25 was considered as the low expression of LHPP, and the total LHPP expression score > 1.25 was considered as the high expression of LHPP. However, in adjacent normal tissues, the total LHPP expression score ≤ 6.25 was considered as the low expression of LHPP, and the total LHPP expression score > 6.25 was considered as the high expression of LHPP [13].

### 2.5. RNA Extraction and qRT-PCR Analysis

Total RNA was extracted from cultured cells or tissues using the Trizol Kit (Invitrogen, Carlsbad, CA, USA). Briefly, 3 mL cell suspension plated into 6-well plates (1 × 10^7^ cells/well) were harvested and washed with cold PBS. Or 50 mg HCC tissues or their adjacent normal tissues were frozen by liquid nitrogen and ground very fine. Subsequently, 1 mL Trizol was added to the harvested cells or ground tissues and maintained 1 min at 4°C for cell lysis. Then, 0.2 mL chloroform was added to lysis and shaken for 15 s. Samples were centrifugated for 15 min at 12000g rpm at 4°C, and supernatant contained total RNA was transferred to a 1.5 mL tube, and add 0.5 ml isopropanol, mix the liquid gently, and let it stand for 10 min at room temperature. And then, samples were centrifugated for 10 min at 12000g rpm at 4°C and the supernatant was discarded. Finally, 100 *μ*L of sterile-filtered water treated with diethyl pyrocarbonate (DEPC) was added to dissolve total RNA.

cDNA was obtained through reverse transcription using the Promega M-MLV Kit (Promega, Madison, WI, USA). Quantitative real-time PCR (qRT-PCR) was performed using the 7500 Real-Time PCR System (ABI, California, USA). The SYBR Master Mixture Kit (Takara, Japan) and RNA reverse transcription were performed to determine expression.

### 2.6. Western Blot Analysis

The cells or tissues frozen by liquid nitrogen and ground were lysed and centrifuged at 12,000g for 15 min at 4°C. Then, total protein was extracted from the resulting supernatant, and the concentration was quantified through the bicinchoninic acid (BCA) assay. Equal amounts (30 *μ*g) of proteins were separated using 10% sodium dodecyl sulfate-polyacrylamide gel (SDS), followed by transfer onto polyvinylidene difluoride membranes. After blocking with defatted milk powder, the membranes were treated with rabbit monoclonal anti-human *β*-actin and LHPP antibodies (1 : 1000 dilution) overnight at 4°C. This was followed by incubation with appropriate HRP-conjugated secondary antibodies at room temperature for 1 h and detected using an enhanced chemiluminescence (ECL) kit (GE Healthcare, Beijing, China).

### 2.7. Detection of AFP and GGT of Blood

The levels of AFP and GGT of blood were detected by enzyme-linked immunosorbent assay (ELISA) using a chemiluminescence immune analysis system (Dxl800Access, Beckman, USA). All procedures were strictly in accordance with the standard operating procedure.

### 2.8. Statistical Analysis

The differential expression of LHPP in HCC tissues and their adjacent normal tissues was evaluated using the nonparametric tests. The survival curves depending on the expression of LHPP and clinical characteristics were drawn by the Kaplan-Meier method and log-rank test. Subsequently, all the potential predictive factors were involved in the Cox multivariate regression survival analysis. The Spearman rank correlation coefficient was used to evaluate the correlation between the expression of LHPP and some clinical immunohistochemical factors. All statistical analyses were conducted using SPSS 17.0 software. *P* < 0.05 was considered significant.

## 3. Results

### 3.1. Participant Characteristics

90 paired HCC and paired adjacent normal tissues were obtained from patients who underwent primary surgery in the Taizhou Hospital of Zhejiang Province (Taizhou, China) between January 2010 and November 2015. In this study, there were 90 participants including 80 males (88.8%) and 10 females (11.2%) and 71(88.7%) with mean age ≤ 60 years. There were 62 (68.9%) patients with tumor size < 5 cm. 58 (64.4%) cases were T1 stage, and patients with clinical Stage I, II, and III were 58 (64.4%), 28 (31.1%), and 4 (4.44%), respectively (Table 1).

### 3.2. Result of Immunohistochemical Analysis

The result of immunohistochemical analysis showed that the expression of LHPP in HCC was significantly downregulated compared with paired adjacent normal tissues (3.63 ± 2.75 vs. 8.63 ± 1.25, *P* < 0.001) (Figure 1(a)). Also, it is found that expressions of LHPP of cytoplasm or cell nucleus in HCC were significantly downregulated than those in paired adjacent normal tissues (Figures 1(b) and 1(c)).

### 3.3. Expressions of mRNA and Protein of LHPP in Tissues and Cells

Relative mRNA levels of LHPP in HCC tissues and paired adjacent samples and cultured cells were examined through qRT-PCR. The results showed relative mRNA levels of LHPP in tumor samples were markedly lower than those of the adjacent normal tissues (Figure 2(a)). Also, relative mRNA levels of LHPP in HepG2, BEL-7404, and SMMC-7721 cell lines were significantly lower than those of LO-2 cells (Figure 2(c)).

Protein levels of LHPP in tissues and cells were detected by Western blot analysis (WB). As showed in Figure 2(b), the protein expression levels of LHPP in HCC tissues were significantly lower than those in the adjacent normal tissues. Additionally, the data showed that the expression of LHPP in HepG2, BEL-7404, and SMMC-7721 cell lines was much lower than that in LO-2 cells (Figure 2(d)).

### 3.4. Correlation of the Expression of LHPP with the Clinical Index of HCC

The expression of LHPP negatively correlated with tumor size in HCC (*r* = 0.303; *P* = 0.005). The nuclear expression of LHPP in paired adjacent normal tissue negatively correlated with tumor size (*r* = 0.261; *P* = 0.023), while the cytoplasmic expression of LHPP in nontumor tissues correlated with vascular invasion (*r* = 0.300; *P* = 0.012) or recurrence (*r* = 0.348; *P* = 0.002). No significant correlation was found between LHPP expression and gender age pathological grading, vascular invasion, T clinical stages, recurrence, or liver cirrhosis (Table 2).

### 3.5. Correlation between the Expression of LHPP and the Expression Levels of GGT and AFP

To further investigate the correlation between the expression of LHPP and the expression levels of LHPP, GGT and AFP were detected in plasma and HCC tissue by ELISA and Spearman's rho test. Results showed that expression of LHPP of the plasma and HCC tissue of patients negatively correlated with GGT and AFP levels in blood and HCC tissues (Table 3).

### 3.6. Correlation between Survival and Expression of LHPP

Correlation between survival and expression of LHPP in HCC cancer or paired adjacent normal tissue was analyzed using the Kaplan-Meier method and the log-rank test. Results showed the overall survival of a patient with higher expression of LHPP and lower expression of LHPP in HCC tissue has no difference statistically (*P* = 0.369) (Figure 3(a)). However, disease-free (DSF) survival of patients with the high expression of LHPP was significantly higher than patients with the low expression of LHPP in HCC tissue (53.4% vs. 25.9%, *P* = 0.012) (Figure 3(b)). The overall survival of patients with the high expression of LHPP was much higher than those with the low expression of LHPP in adjacent normal tissue (71.7% vs. 31.3%, *P* = 0.004) (Figure 3(c)). Also, it was found DSF survival of patients with the high expression of LHPP was markedly higher than those with the low expression of LHPP in adjacent normal tissue (55.0% vs. 12.5%, *P* = 0.008) (Figure 3(d)).

## 4. Discussion

Histidine phosphorylation, also known as the hidden phosphoproteome, is a poorly characterized posttranslational modification of proteins. LHPP is a protein histidine phosphatase and a tumor suppressor, suggesting that deregulated histidine phosphorylation is oncogenic [6]. A previous study suggested that LHPP acted as a tumor suppressor in various cancers, such as hepatocellular carcinoma, cervical cancer, bladder cancer, pancreatic cancer, and melanoma. In hepatocellular carcinoma (HCC), decreased expression of LHPP is positively correlated with larger tumor size and reduced overall survival [11]. But the correlation between the expression of LHPP and the clinical parameters of oncogenic progression is not fully studied.

In this study, the Spearman rank correlation coefficient was used to evaluate the correlation of the expression of LHPP and the clinical index of HCC. Results showed that LHPP expression in HCC was correlated with tumor size, indicating the potential function of LHPP on tumor proliferation. The expression of LHPP in paired adjacent normal tissue significantly negatively correlated with vascular invasion and recurrence. A comparison of the expression of LHPP in HCC tissues and their paired adjacent normal tissue suggested that the expression of LHPP in HCC and adjacent normal tissue might inhibit the progression of HCC *via* different mechanisms.

AFP and GGT, as two important HCC markers, have clinical significance in the diagnosis of HCC [14, 15]. To further investigate the role of LHPP in HCC, the expression levels of GGT and AFP were detected in the blood and tissue. Spearman's rho test results showed that expression of LHPP of the plasma and HCC tissues of patients negatively correlated with GGT and AFP levels. The present study validated that the expression of LHPP correlated with the expression of AFP and GGT in blood and HCC tissue, suggesting that LHPP correlated with the incidence of HCC or served as a complementary biomarker for AFP and GGT in diagnosing HCC.

LHPP gene variation is associated with the oral cavity and pharyngeal cancer [9]. In this study, the results of HCC microarray showed that the expression of LHPP was the lowest in HCC tissue, with lower expression in primary liver cancer and higher expression in paired adjacent normal tissue, illustrating that LHPP might inhibit the distant metastasis of HCC. The present study demonstrated that LHPP could inhibit the progression and the distant metastasis of HCC. As metastasis has been reported a leading cause of cancer-related death [11], it was speculated that the expression of LHPP was associated with tumor severity, and LHPP could act as a tumor suppressor.

The Kaplan-Meier method and the log-rank test were employed to reveal the correlation between the expression of LHPP in HCC tissue or adjacent normal tissue and the prognosis of HCC. Results showed DSF survival of patients with the high expression of LHPP was significantly higher than patients with the low expression of LHPP in HCC tissue. Also, it was verified that overall survival and DSF survival of patients with the high expression of LHPP were markedly higher than those with the low expression of LHPP in paired adjacent normal tissue.

Our study suggests that LHPP plays an important role in the occurrence and development of HCC and provides a potential marker of HCC. However, due to the limited number of samples, whether it can be used as an occurrence and development marker of HCC and as a diagnostic indicator of HCC needs further study.

## 5. Conclusions

The present study has validated there was a significant differential expression of LHPP in HCC tissues and their paired adjacent normal tissue. It is suggested that the expression of LHPP was associated with the AFP level and good prognosis in HCC, and LHPP is expected to be a potential marker of HCC.

## Figures and Tables

**Figure 1:** Expression of LHPP in the nucleus and plasma of tumor and normal samples. Expressions of LHPP in 90 liver cancer and paired adjacent normal tissue were detected through immunohistochemical staining, and staining intensities were calculated for immunohistochemical analysis. (a) Representative immunohistochemical images of the expression of LHPP in tumor and adjacent normal tissue. (b) Cytoplasmic expression of LHPP in tumor and adjacent normal tissue. (c) Nuclear expression of LHPP in tumor and adjacent normal tissue. ^∗∗∗^*P* < 0.001 vs. the corresponding control.

**Figure 2:** Expressions of mRNA and protein of LHPP in tissues and cells *in vitro*. (a) Relative mRNA levels of LHPP in cancer and paired adjacent normal tissue. Total RNA of 5 liver cancer and adjacent normal tissue were extracted, and relative mRNA levels of LHPP were examined through qRT-PCR. (b) Relative protein expressions of LHPP in cancer and paired adjacent normal tissue. Total protein of 5 liver cancer and adjacent normal tissue was extracted, and protein expressions of LHPP were examined through WB. (c) Relative mRNA levels of LHPP in HepG2, BEL-7404, SMMC-7721, and LO-2 cell lines. Total RNA of HepG2, BEL-7404, SMMC-7721, and LO-2 cells were extracted, and relative mRNA levels of LHPP were examined through qRT-PCR. (d) Relative LHPP expressions in HepG2, BEL-7404, SMMC-7721, and LO-2 cell lines. Total protein of HepG2, BEL-7404, SMMC-7721, and LO-2 cell lines was extracted, and protein expressions of LHPP were examined through WB. ^∗^*P* < 0.05 and ^∗∗^*P* < 0.01 vs. the corresponding control.

**Figure 3:** Correlation of survival and expression of LHPP in HCC tissue and paired adjacent normal tissue. Immunohistochemical analysis was employed to detect the differential expression of LHPP in HCC tissues or paired adjacent normal tissue, and the Kaplan-Meier method and the log-rank test were used to analyze the correlation of survival and expression of LHPP. (a) Correlation of overall survival and expression of LHPP in HCC tissue. (b) Correlation of disease-free survival and expression of LHPP in HCC tissue. (c) Correlation of overall survival and expression of LHPP in adjacent normal tissue. (d) Correlation of disease-free survival and expression of LHPP in paired adjacent normal tissue. ^∗^*P* < 0.05 vs. the corresponding control.

**Table 1:** The HCC patients' clinical information in detail.

	Clinical index	*N*	Total *N*
Gender	Male	80	90
	Female	10	

Age	≤60 years	71	90
	>60 years	19	

Tumor size	≤5 cm	62	90
	>5 cm	28	

T staging	T1	58	90
	T2-T3	32	

Clinical staging	Stage I	58	90
	Stage II	28	
	Stage III	4	

**Table 2:** Correlation of the expression of LHPP and the clinical index of HCC.

			Gender	Age	Pathological grading	Tumor size	Tumor number	Cirrhotic nodule	Tumor cell membrane	Vascular invasion	T	Clinical stages	Recurrence	Liver cirrhosis
Spearman's rho	LHPP expression in the nucleus of HCC	Correlation coefficient	0.019	-0.033	0.057	-0.274^∗^	0.175	0.202	-0.064	-0.007	0.075	0.075	-0.056	-0.023
		Sig. (2-tailed)	0.874	0.776	0.626	0.017	0.130	0.082	0.585	0.954	0.518	0.518	0.633	0.845
		*N*	76	76	76	76	76	75	75	70	76	76	76	75
	LHPP expression in adjacent normal tissue	Correlation coefficient	-0.079	0.013	-0.108	-0.241^∗^	0.150	0.163	-0.010	-0.116	-0.053	-0.053	-0.181	0.089
		Sig. (2-tailed)	0.497	0.910	0.354	0.036	0.196	0.163	0.932	0.338	0.650	0.650	0.117	0.446
		*N*	76	76	76	76	76	75	75	70	76	76	76	75

^∗^Correlation is significant at the 0.05 level (2-tailed).

**Table 3:** The relationship between the expression of LHPP and the GGT and AFP expression levels in blood and HCC tissues.

				HBsAg	HBcAb	TB	ALT	ALB	AFP	GGT	PTT
Spearman's rho	LHPP level in the plasma	Patients	Correlation coefficient	-0.027	-0.069	0.196	-0.033	0.114	-0.063	0.044	0.053
			Sig. (2-tailed)	0.808	0.536	0.075	0.763	0.301	0.571	0.691	0.630
			*N*	84	82	84	84	84	84	84	84
		Normal	Correlation coefficient	-0.017	0.187	-0.046	-0.144	0.111	-0.150	-0.269^∗^	-0.174
			Sig. (2-tailed)	0.882	0.113	0.692	0.219	0.342	0.200	0.020	0.136
			*N*	75	73	75	75	75	75	75	75
	LHPP expression in the tissues	Tumor	Correlation coefficient	0.035	0.022	0.039	-0.042	-0.052	-0.232^∗^	0.047	0.185
			Sig. (2-tailed)	0.766	0.851	0.738	0.720	0.655	0.045	0.686	0.112
			*N*	75	73	75	75	75	75	75	75
		Paratumor	Correlation coefficient	-0.117	0.147	0.062	-0.223	0.093	-0.121	-0.193	-0.142
			Sig. (2-tailed)	0.317	0.216	0.599	0.054	0.426	0.300	0.097	0.223
			*N*	75	73	75	75	75	75	75	75

^∗^Correlation is significant at the 0.05 level (2-tailed).

## Data Availability

Dataset can be accessed from the corresponding author upon reasonable request.
